This article has been retracted.

# Appraisal of foliar spray of iron and salicylic acid under artificial magnetism on morpho-physiological attributes of pea (*Pisum sativum* L.) plants

**DOI:** 10.1371/journal.pone.0265654

**Published:** 2022-04-14

**Authors:** Hassan Naseer, Kanval Shaukat, Noreen Zahra, Muhammad Bilal Hafeez, Ali Raza, Mereen Nizar, Muhammad Akram Qazi, Qasim Ali, Asma A. Al-Huqail, Manzar H. Siddiqui, Hayssam M. Ali

**Affiliations:** 1 Department of Botany, University of Balochistan, Quetta, Pakistan; 2 Department of Botany, University of Agriculture, Faisalabad, Pakistan; 3 Department of Agronomy, University of Agriculture, Faisalabad, Pakistan; 4 Fujian Provincial Key Laboratory of Crop Molecular and Cell Biology, Oil Crops Research Institute, Center of Legume Crop Genetics and Systems Biology/College of Agriculture, Fujian Agriculture and Forestry University (FAFU), Fuzhou, China; 5 Directorate of Soil Fertility Research Institute, Lahore, Pakistan; 6 Institute of Food and Agriculture Sciences, University of Florida, Gainesville, Florida, United States of America; 7 Department of Botany and Microbiology, College of Science, King Saud University, Riyadh, Saudi Arabia; National University of Kaohsiung, TAIWAN

## Abstract

The appraisal of foliar treatment of iron (Fe) and salicylic acid (SA) on plant under artificial magnetism is very crucial in understanding its impact on growth and development of plants. The present study was designed to document the potential role of Fe and SA on pea (*Pisum sativum* L.) Matore variety exposed to different magnetism treatments (geomagnetism and artificial magnetism). Thus a pot experiment was conducted using Completely Randomized Design under factorial with three replicates. Various artificial magnetic treatment were applied in pots prior to sowing. Further, 15 days germinated pea seedlings were foliarly supplemented with 250 ppm Fe and 250μM SA, moreover after 20 days of foliar fertilization plants were harvested to analyze and record various morpho-physiological attributes. Data elucidate significant variations in pea plants among different treatments. Artificial magnetism treatments in combination with foliar application of Fe and SA significantly improved various growth attributes (root and shoot length, fresh and dry weights of root and shoot, leaf area), photosynthetic pigments (Chl *a*, *b* and carotenoids) and the contents of soluble sugars. However, oxidative stress (H_2_O_2_ and MDA) enhanced under different magnetism treatment but foliar application of Fe and SA hampered the production of reactive oxygen species thereby limiting the concentration of H_2_O_2_ and MDA in plant tissues. Furthermore the accumulation of nutrients (iron, potassium and nitrate) profoundly increased under artificial magnetism treatment specifically under Fe and SA foliar treatment excluding nitrate where Fe foliar treatment tend to limit nitrate in plant. Consequently, the present research interestingly highlights progressive role of Fe and SA foliar treatment on pea plants under artificial magnetism. Thus, foliar supplementation may be suggested for better growth and development of plants combined with magnetic treatments.

## 1. Introduction

Green pea or field pea (*Pisum sativum* L.) is a member of the Fabaceae family (legumes), an important family of angiosperms. It is an annual cold season crop grown in almost every part of the world [1]. Legumes consist of pre-annual and annual herbs, most of which are important economically as well as nutritionally. These legumes serve as store house of protein for both humans and animals, and these also increase soil fertility with nitrogen-fixing bacteria [2]. Germination of pea seeds can be increased by pre-sowing treatments bringing chemical and physical changes by breaking dormancy which protects the seeds against biotic, abiotic stress, diseases, and pests and gives uniformity in the establishment of crops in the field [3]. Hettiarachchi et al. [4] reported *TOP2* expression (Topoisomerase II) in pea plant gets upregulated under various abiotic stresses such as salinity and chilling stress.

The change in the living environment due to the magnetic field is very crucial. Due to the effects of magnetic fields, various changes induces in development and growth of living organisms. Plants are indeed the best model to study the biological effects of magnetic fields [5]. Electromagnetic treatment effects on various plants are well documented in various studies with remarkable findings, especially under various abiotic stresses; drought [6], salinity [3], and temperature [7]. Seed germination gets stimulated under an optimal electromagnetic field [8]. The magnetic field increases seed energy and disperses the energy to biomolecules that stimulate the metabolism, thereby increasing germination [8]. Magnetic and electric treatments tend to improve seed vigor, improve seed germination and growth by stimulating the activity of proteins, and enhance antioxidant enzymes [9–11]. Khade and Mancharkar [12] documented that various research has shown positive effects of electromagnetic fields on germination and growth of selected varieties of beans noting improvement in germination parameters and higher yield. Mahajan and Pandey [13] noted that pretreatment of seed with static magnetic field 226 mT millitesla for 100 min increased germination rate and decreased malondialdehyde (MDA), hydrogen peroxide (H_2_O_2_), and superoxide (O_2_^-^) in *Vigna radiata* [3] also stated that seed priming at 200 mT increased α-trocopherol and ascorbic acid contents while decreased H_2_O_2_ in soybean. Furthermore, magnetic pre sowing treatments of seeds allow to reduce the cost of planting as germination rates improves [13]. Moon and Chung [14] documented that magnetic field has significant effect on seed germination of tomato. In another study, Ul-Haq et al. [15] stated that physical pre-sowing activities such as growing seeds with magnetism are much more nature friendly, secure, and much more inexpensive than chemicals. It also increases the free movement of ions and radicals in the soil without damaging the soil organic matter and also have no detrimental effects on seed profile hence results in healthier and uniform crop stands.

Plant growth regulators have shown to positively influence seed germination of various plant species. Many crops such as soybeans, peas, corn, and small grains have very less dormancy period after seed maturity. Seed dormancy is stimulated by gibberellins [16]. Gibberellin is involved in many important biological functions of plants such as plant height, cell division, leaf expansion, elongation, photosynthesis, transpiration rate and in flowering [17]. Changing the metabolism of some plant species like peas with plant growth regulators to control the disease has shown varying results. Salicylic acid in recent years became the key interest phytohormone as it has been designated to be endogenous regulatory signal mediating defense response to various abiotic stresses; heat [18], drought [19], osmotic stress [20], heavy metal [21], and chilling [22]. Moreover it play fundamental role in local and systemic response under biotic stress [23].

Salicylic acid (SA), also known as 2_hydroxy benzoic acid, is the most diverse group of phenolic compounds consisting of an aromatic ring having a hydroxyl group as a functional group that is biosynthesized by plants. SA induces tolerance in plants by mediating signal transduction in plants against abiotic stress [24, 25]. SA when applied foliarly increases contents of peroxidase (POD), superoxide dismutase (SOD), catalase (CAT), soluble sugars, glycine betaine, protein, relative water content (RWC), root and leaf K^+^ while decreased Na^+^, H_2_O_2_, O_2_^•−^, and MDA contents [26]. SA priming increases total soluble sugars, proline, and indole acetic acid while decreases gibberellins, abscisic acid, and total soluble protein [27]. Moreover, Yadav et al. [28] reported an increase in plant height and grain yield of wheat with better RWC%, total Chl contents, and Fluorescence variable/ Fluorescence maximum with SA foliar supplementation under salinity and drought stress; however membrane injury and lipid peroxidation get hampered thus validating the defensive role of SA. Additionally, SA positively or negatively correlates with other plants regulators to help plants and to protect plants against pathogen attack [29].

Iron (Fe) is 4^th^ most abundant element on the earth and found in the crystal lattices of most minerals [30]. Fe in plants is mostly in Fe (III) form and very less in Fe (II) form, and most of the Fe about 90% found in chloroplast and particularly in chloroplasts of those leaves which undergo rapid growth [31]. Soil quality is very vital for plant growth and development. Deficiency of Fe could lead to calcareous soil conditions, whereas high concentration of Fe in soil could lead to waterlogging soil conditions [32]. Due to deficiency of Fe in plants chlorosis occurs in leaves that results in decreased translocation of photosynthates [33], limited accumulation of total biomass, reduced growth of root and shoot, and leaf area [34]. However, when there is an excess Fe in plants, it can cause brown spots on leaves, reduced efficiency of photosystem II and decreased rate of photosynthesis [35]. Literature documents that exogenous supplementation of Fe increases growth and yield of crops [36–38]. Although vast literature exists regarding magnetic treatment and impact of foliar supplementation of SA and Fe but no research has yet been reported on the combined effect of the two factors (magnetism and foliar supplementation). Present study was conducted to evaluate the influence of geo and artificial magnetism on seedling growth of *Pisum sativum* L. and to determine the possible role of foliarly applied SA and Fe in improving seedling growth in response to magnetism.

## 2. Materials and methods

### 2.1. Study area

Study area of this research is Quetta which is the capital city of province Balochistan, Pakistan. Quetta is situated at 1679 meters above sea level. Whereas the climate of the Quetta is quite cold and semi-arid. The temperature of Quetta is very diverse between summers to winter. The average rain fall is less than 250 mm per year. While June and July are the warmest months of the year where the temperature ranges from 35°C to 40°C. January is the coolest month of the year when the temperature ranges from 11°C to -7°C or less. For the experiment, seeds of Matore variety of *Pisum sativum* were taken from the Agriculture Department, Mastung road Quetta. The experiment was conducted in the Botanical Garden University of Balochistan, Quetta.

### 2.2. Experiment layout

A pot experiment was conducted in the prevailing environmental conditions of Quetta. The experimental design was completely randomized under factorial with three replicates. Pots of 32 cm diameter were filled with 8 kg of soil from Agriculture Department Quetta. The soil ratio was taken as 60:20:20., i.e., soil, sand, and manure, respectively. Seeds were sown at 1 inch depth. Five seeds were sown in each pot. Different treatments of artificial magnetism were applied prior to the sowing of the seeds in comparison to geo magnetism treatment (no external magnet placed). Treatment includes Geo Magnetism; Artificial Magnetism that includes;magnet South (S) root, magnet North (N) root, S root/ N shoot, N root/ S shoot, N/S root and S/N shoot, S/N root and N/S shoot under complete set of; no foliar spray (Control conditions/ control set/ control), Fe 250 ppm and SA 250 μM spray. Thus a total 63 pots was used. The foliar concentration were selected on preliminary trials, and thus one the most suitable level was selected for the present research. After 15 days of seed germination, selected level of SA and Fe were foliarly applied to both the sets (i.e., geo and artificial magnetism treated plants). After 20 days of foliar spray, plants were harvested, and data was collected regarding various morpho-physiological attributes.

### 2.3. Growth parameters

Length of shoot and root were measured in centimeters using scale. Leaves of plants were counted/plant each treatment. Leaf area per plant was calculated using the formula (LxW x A¼ 0.75). Here L denotes the length of the leaf, W denotes the width of the leaf, and 0.75 is a correction factor. Formula developed by Cain and Castro [39]. After harvest, plant fresh shoot and root weight were obtained immediately. Dried weight of shoot and root were taken after samples were dried into the oven at 65°C -75°C.

### 2.4. Physiological and biochemical analysis

#### 2.4.1. Photosynthetic pigment analysis

For the analysis of photosynthetic pigments, 0.1 g of leaf sample was taken and grinded in 1–2 ml of 80% acetone, maintained volume upto 10mL, using 80% acetone. Absorbance was noted at 663, 645, and 480 nm against 80% acetone as blank. The chlorophyll calculation was done using the formula of Arnon [40].


$$\text{Chlorophyll},\;\text{a}\left(\text{mg}/\text{g}\;\text{FWT}\right)=\left(1.27\times \text{A}663-2.69\times \text{A}645\right)\;\text{V}/1000\times \text{W}$$

$$\text{Chlorophyll},\;\text{b}\left(\text{mg}/\text{g}\;\text{FWT}\right)=\left(22.9\times \text{A}645-4.68\times \text{A}663\right)\;\text{V}/1000\times \text{W}$$

#### 2.4.2. Carotenoid analysis

Calculation of carotenoids analysis was done following Kirk [41] formula

$$\left(\text{A}480+0.114.\;\text{A}663-0.638\times \text{A}645\right)/2500\;\text{X}\;1000).$$

Where A480, A645, and A663 are the absorbance of the acetone extract at 480 nm, 645nm, and 663 nm, respectively.

V = Acetone extract volume.

W = Leaf weight (gram fresh weight.).

#### 2.4.3. Soluble sugars

Soluble sugars was measured according to Yoshida et al. [42]. Plant sample of 0.1 g was taken and boiled in 5 mL of the distilled water in water bath for about 1 hour. From the extract, 1 mL was taken, followed by adding 9 mL of distilled water for dilution. From this extract, 0.5 mL was taken and added 5mL of anthrone reagent. After Vortex, the mixture and was kept in water bath at 90°C for about 20 minutes. The absorbance was taken at 620nm by using spectrophotometer. Distilled water was used as a blank.

#### 2.4.4. Hydrogen peroxide (H_2_O_2_)

Fresh plant samples (0.1g) were grinded in 2 mL of 0.1% (w/v) trichloroacetic acid (TCA) under pre-chilled conditions by crushing the tissues (Placed on ice bath). The homogenized material was then centrifuged at 12000 rpm for 15 min. The supernatant (0.5 mL) was mixed with 0.5 mL of potassium phosphate buffer (pH 7.0), and 1 mL of potassium iodide solution, thoroughly mixed, and absorbance was recorded at 390 nm. Distilled water was used as blank Velikova et al. [43].

#### 2.4.5. Malondialdehyde (MDA)

Malondialdehyde was determined by the method developed by Heath and Packer [44]. Plant sample (0.1 g) of plant fresh material was grinded in 1 mL of (1% w/v) TCA and centrifuged at 12,000 rpm for 15 minutes. After that, 1mL of supernatant was taken and mixed with 1 mL of 0.5% thiobarbituric acid in 20% TCA [0.5% in 20% (w/v) TCA] and kept in a water bath preheated at 95°C for 50 minutes. The sample extract was cooled in an ice bath. Absorbance was measured at 532 nm and 600 nm. For comparison, 1% TCA was used as blank. MDA contents were calculated using its absorption coefficient of 155000 nmol/mol as:

$$\text{MDA}\;(\text{nmol}\;{\text{mL}}^{-1}=\left[\left(\text{A}532-\text{A}\;600\right)/155000\right]10^{6}$$

### 2.5. Nutrients analysis

Nutrient analysis was done to evaluate the differences among treatments such as nitrate, Fe, and potassium.

#### 2.5.1. Nitrate

The oven-dried plant samples were digested using nitric acid and diluted with distilled water up to 30mL. From the digested sample, 3ml of the extract was taken, and 7ml of CTA (Chromo tropic acid) was added and was left for 20 minutes. Absorbance at 430nm was measured according to the method developed by Kowalenko and Lowe [45].

#### 2.5.2. Determination of iron and potassium

Determination of iron and potassium in plant samples were determined by using atomic absorption spectrophotometer Yoshida et al. [42].

### 2.6. Statistical analysis

Statistical analysis was performed using “STATISTIX 8.1”. Graph, mean and standard deviation were calculated using MS.EXCEL.

## 3. Results

### 3.1. Morphological parameters

#### 3.1.1. Root length

Data regarding the root length of *Pisum sativum* revealed significant differences (P<0.05) among different treatments (Fig 1A). Highest root length was observed when plant was given South magnet to root under control conditions (No foliar spray) while least root length was observed when plant was given S root / N shoot treatment under control conditions (Fig 1A). South Root magnetic treatment increased root length upto 63.41% in comparison to geomagnetism.

**Fig 1:** Effect of different magnetic treatments on the Morphological Attributes; Root length (A), Shoot length (B), No of leaves plant^-1^ (C), Leaf area (D) Root fresh weight (E), shoot fresh weight (F) Root dry weight (G), shoot dry weight (H) of *Pisum sativum* in response to Fe and SA Foliar Spray. The same letters on graphs represent statistically similar effect (P<0.05).

The data trend of root length of pea plant under artificial / geo magnetism treatments and different foliar spray is as follows: S root + control conditions > N root / S shoot + control condition > S root / N shoot + iron foliar spray > N/S root and S/N shoot + iron foliar spray > S root + SA foliar spray > N root SA foliar spray > S/N root and N/S shoot + iron foliar spray > S root + iron foliar control condition > N/S root and S/N shoot + control condition > S root/ N shoot + SA foliar spray > N root + iron foliar spray > N root / S shoot + SA foliar spray > N/S root and S/N shoot + SA foliar spray > S/N root and N/S shoot + control condition > S/N root and N/S shoot + SA foliar spray > geo magnetism + SA foliar spray > N root / S shoot + iron foliar spray > S root / N shoot + control condition.

To wrap up the above results for root length it was noted that root length of pea plant increased under different artificial magnetism treatment in control condition (no foliar spray) and Fe foliar spray whereas SA foliar application was least effective (Fig 1A).

#### 3.1.2. Shoot length

As far as data of shoot length is concerned, it showed statistically significant results (P<0.05). Maximum shoot length was recorded in N/S root and S/N shoot treated plants under Fe foliar spray whereas minimum shoot length was recorded under S root / N shoot treatment with SA foliar spray (Fig 1B). An increase of 35.29% was observed in South Root treatment (control condition) and 52.41% in N/S Root and S/N Shoot magnet treatment (SA spray) over respective geomagnetism treatment.

Data trend of shoot length of *Pisum sativum*, under different foliar spray and artificial / geo magnetism is as follows: N/S root and S/N shoot + Fe foliar spray > N root + control condition > S root + Fe foliar spray > S root + control > N root / S shoot + control condition > S root + Fe foliar spray > N root + Fe foliar spray > geo magnetism + Fe foliar spray > S/N root and N/S shoot + control condition > S/N root and N/S shoot + Fe foliar spray = geo magnetism + control condition > N/S root and S/N shoot + SA foliar spray > S/N root and N/S shoot + SA folia spray > N/S root and S/N shoot + control condition > S root / N shoot + Fe foliar spray > geo magnetism + SA foliar spray > N root / S shoot + SA foliar spray > N root + SA foliar spray > S root / N shoot + control condition > N root / S shoot + Fe foliar spray = S root / N shoot + SA foliar spray.

Considering overall results of shoot length it was observed that treatment of different artificial magnetism had positive impact on shoot length of pea plant as it enhanced the shoot length except for S Root/ N Shoot magnetic treatment where even the impact of Fe and SA foliar treatment seems to be nullified; as this treatment had the shortest plants as compared to all other treatments (Fig 1B).

#### 3.1.3. Number of leaves plant^-1^

Data regarding of number of leaves per plant showed statistically significant results (P<0.05). Highest number of leaves was observed under S/N root and N/S shoot magnetism treatment control conditions however minimum number of leaves were observed under S root / N shoot magnetism with SA foliar spray (Fig 1C). North magnet treatment alone or in combination tend to increase number of leaves upto 40% in comparison to geomagnetism (under absence of foliar treatment).

As far as data of number of leaves plant^-1^ is concerned, trend of data observed is as follows: S/N root and N/S shoot + control condition > N/S root and S/N shoot + control condition > geo magnetism + control condition > N root + control condition = N/S root and S/N shoot + Fe foliar spray > S/N root and N/S shoot + Fe foliar spray > geo magnetism + Fe foliar spray > N root / S shoot + control condition > N root + Fe foliar spray > S root + control condition > S root / N shoot + Fe foliar spray > N root + SA foliar spray > S root + SA foliar spray > S root + Fe foliar spray = S/N root and N/S shoot + SA folia spray > S root / N shoot + control condition > geo magnetism + SA foliar spray > N root / S shoot + Fe foliar spray = N root/ S shoot + SA foliar spray = N/S root and S/N shoot + SA foliar spray > S root / N shoot + SA foliar spray.

In a nutshell, considering the results of number of leaves plant^-1^ it was observed that absence of foliar treatment (Control set) had greater number of leaves plant^-1^ in almost all magnetic treatments as compared to the foliarly supplemented plants (Fig 1C).

#### 3.1.4. Leaf area plant^-1^

Data of leaf area plant^-1^ revealed that data was statistically significant (P<0.05). Maximum leaf area was noted under North Root magment treatment control condition whereas minimum leaf area was noted when plant was given S root / N shoot treatment with SA foliar application (Fig 1D). An increase of 64.82% was observed in South Root magnetic treatment (control condition) over geomagnetism treatment.

The data of leaf area plant^-1^ of *Pisum sativum* revealed following trend under different foliar spray and artificial / geo magnetism treatments: N root + control condition > N root + iron foliar spray > S root + control condition > geo magnetism + iron foliar spray > S root + SA foliar spray > geo magnetism + control condition > N/S root and S/N shoot + iron foliar spray > N/S root and S/N shoot + SA foliar spray > S root + iron foliar spray > S root / N shoot + control condition > S/N root and N/S shoot + iron foliar spray > N root + SA foliar spray > N/S root and S/N shoot + control condition > N root / S shoot + iron foliar spray > N root/ S shoot + control condition > S/N root and N/S shoot + control condition > S/N root and N/S shoot + SA foliar spray > geo magnetism + SA foliar spray > S root / N shoot + iron foliar spray > N root / S shoot + SA foliar spray > S root/ N shoot + SA foliar spray.

Overall results of leaf area plant^-1^ revealed that Fe foliar spray application tend to enhance the leaf area especially under geomagnetism treatment; however, SA foliar spray was least effective in almost all artificial magnetic treatments (Fig 1D).

#### 3.1.5. Root fresh weight

Data of root fresh weight (RFW) of *Pisum sativum* revealed statistically significant results among different treatments (P<0.05). Highest root fresh weight was observed under South Root magnetism with SA foliar application, while least root fresh weight was noted under S root / N shoot magnetism with Fe foliar application (Fig 1E). South Root magnetic treatment in comparison to geomagnetism tend to increase RFW several folds under SA foliar treatment but tend to decrease (34.94%) in absence of any foliar treatment.

The trend of root fresh weight under artificial / geo magnetism and different foliar spray is as follows: S root + SA folia spray > N/S root and S/N shoot + Fe foliar spray > N root + SA foliar spray > geo magnetism + control condition > S/N root and N/S shoot + SA foliar spray > N root + control condition > S root + Fe foliar spray > S root / N shoot + SA foliar spray > N/S root and S/N shoot + SA foliar spray > N root / S shoot + SA foliar spray > geo magnetism + Fe foliar spray > S/N root and N/S shoot + Fe foliar spray > N root / s shoot + control condition > S root + control condition > N/S root and S/N shoot + control condition > N root / S shoot + Fe foliar spray > S/N root and N/S shoot + control condition > S root / N shoot + control condition > N root + Fe foliar spray > geo magnetism + SA foliar spray > S root / N shoot + Fe foliar spray.

Concludingly, considering the root fresh weight of *Pisum sativum* it was noted that SA foliar spray enhanced root fresh weight under almost all artificial magnetism treatment (Fig 1E).

#### 3.1.6. Shoot fresh weight

Data for shoot fresh weight (SFW) showed statistically significant results (P<0.05). Maximum shoot fresh weight was observed in plants under North Root treatment under control condition, whereas minimum shoot fresh weight was observed under N root/S shoot magnetism with SA foliar application (Fig 1F). SFW tend to decrease 28.18% and 8.78% with South Root magnetism treatment under control and Fe foliar treatment respectively, in comparison to the Pea plants under geomagnetism treatment.

Considering the data of SFWof pea plant, following trend under different foliar spray and artificial / geo magnetism treatments was observed: N root + control condition > geo magnetism + control condition > S root + control condition > S root + SA foliar spray > S root / N shoot + control condition > N root / S shoot + control condition > S/N root and N/S shoot + control condition > S/N root and N/S shoot + iron foliar spray > N/S root and S/N shoot + iron foliar spray > N/S root and S/N shoot + SA foliar spray > S root + iron foliar spray > geo magnetism + SA foliar spray > N/S root and S/N shoot + SA foliar spray > geo magnetism + iron foliar spray > N root /S shoot + iron foliar spray > S root / N shoot + iron foliar spray > N root + SA foliar spray > N root + iron foliar spray > S/N root and N/S shoot + SA foliar spray > S root / N shoot + SA foliar spray > N root / S shoot + SA foliar spray.

Analyzing the overall results of shoot fresh weight it was revealed that pea plants without foliar treatment had greater shoot fresh weight in almost all artificial as well geomagnetism treatment (Fig 1F).

#### 3.1.7. Root dry weight

As far as data of root dry weight (RDW) of *Pisum sativum* is concerned, it was found to be statistically significant (P<0.05) (Fig 1G). Maximum root dry weight was noted under geomagnetism with Fe foliar spray treatment; however, the least root dry weight was recorded under N/S root and S/N shoot treatment with SA foliar spray (Fig 1G). RDW tend to reduce several folds in almost all magnetic treatments in comparison to plants under geomagnetism.

Data trend regarding root dry weight of *Pisum sativum* show following order: Geo magnetism + Fe foliar spray > S/N root and N/S shoot + SA foliar spray > N root / S shoot + SA foliar spray > geo magnetism + SA foliar spray > S root + SA foliar spray > N root / S shoot + control condition > geo magnetism + control condition > S/N root and N/S shoot + Fe foliar spray > N/S root and S/N shoot + Fe foliar spray > S root / N shoot + Fe foliar spray > S root / N shoot + SA foliar spray > S root / N shoot + control condition > N root + control condition > N root + SA foliar spray > S root + control condition > N root / S shoot + Fe foliar spray > N root + Fe foliar spray > S root + Fe foliar spray > N/S root and S/N shoot + SA foliar spray > N/S root and S/N shoot + control condition > S/N root and N/S shoot + control condition.

To wrap up the overall results of root dry weight of pea plant, foliar supplementation of Fe and SA under different magnetism treatment were quite beneficial as root dry weight increased under foliar treatment specifically SA supplementation thus illustrating its positive impact. However, plants under geomagnetism treatment irrespective of foliar treatment had greater RDWs (Fig 1G).

#### 3.1.8. Shoot dry weight

Data regarding shoot dry weight (SDW) of pea plant revealed statistically significant results among different treatments (P<0.05). Maximum shoot dry weight was observed under geomagnetism with Fe foliar spray treatment, whereas minimum shoot dry weight was observed under S/N root and N/S shoot magnetism control conditions (Fig 1H). Similar to RDW, SDW tend to reduce several folds in almost all magnetic treatments in comparison to plants under geomagnetism.

The data of shoot dry weight of pea plant revealed the following trend under different foliar spray and artificial / geo magnetism: Geo magnetism + iron foliar spray > geo magnetism + SA foliar spray > S root + iron foliar spray > S/N root and N/S shoot + iron foliar spray > N/S root and S/N shoot + iron foliar spray > S root + SA foliar spray > S root / N shoot + iron foliar spray > N root + iron foliar spray > S root + control condition > geo magnetism + control condition N root / S shoot + iron foliar spray > S root / N shoot + control condition > N/S root and S/N shoot + SA foliar spray > S/N root and N/S shoot + SA foliar spray > S root / N shoot + SA foliar spray > N root / S shoot + SA foliar spray > N/S root and S/N shoot + control condition > N root / S shoot + control condition > N root + SA foliar spray > N root + control condition > S/N root and N/S shoot + control condition.

Overall results of shoot dry weight of pea plant were quite similar to those of root dry weight. Nonetheless plants under geomagnetism treatment had greater biomass irrespective of foliar treatment (Fig 1H).

### 3.2. Photosynthetic pigments

#### 3.2.1. Chlorophyll *a*

Considering data for chlorophyll *a* (Chl *a*) of pea plant, it showed statistically significant results among different treatments (P<0.05). Maximum chlorophyll *a* was recorded with North Root magnetism under control condition, while minimum chlorophyll *a* was recorded under North root magnetism with SA foliar application (Fig 2A).

**Fig 2:** Effect of different magnetic treatments on the Photosynthetic Pigments; Chlorophyll *a* (A), Chlorophyll *b* (B), Carotenoids (C) of *Pisum sativum* in response to Fe and SA Foliar Spray. The same letters on graphs represent statistically similar effect (P<0.05).

The trend of data for Chl *a* in *Pisum sativum* leaves under artificial / geo magnetism and different foliar spray is as follows: N root + control condition > N/S root and S/N shoot + iron foliar spray > N/S root and S/N shoot + SA foliar spray > geo magnetism + control condition > N root + iron foliar spray > S root + SA foliar spray > N root / S shoot + control condition > S/N root and N/S shoot + SA foliar spray > S root + iron foliar spray > S root + control condition > S root / N shoot + iron foliar spray > N/S root and S/N shoot + control condition > N root / S shoot + iron foliar spray > S root / N shoot + SA foliar spray > geo magnetism + iron foliar spray > N root / S shoot + SA foliar spray > S root / N shoot + control condition > S/N root and N/S shoot + iron foliar spray > S/N root and N/S shoot + control condition > geo magnetism + SA foliar spray > N root + SA foliar spray.

Summing up the results for Chl *a* of *Pisum sativum*, it was observed that SA, and Fe foliar applications under different artificial magnetism treatments had a quite positive impact in improving Chl *a* contents (Fig 2A).

#### 3.2.2. Chlorophyll *b*

Data of chlorophyll *b* (Chl *b*) of pea plant also showed statistically significant results (P<0.05). Maximum Chl *b* was observed under North root magnetism with SA foliar spray, whereas least Chl *b* was noted under geomagnetism with Fe foliar spray (Fig 2B). North Root magnetism treatment tend to increase Chl *b* content 8–43% under Fe and SA foliar treatment.

Considering data trend for Chl *b* in leaves of *Pisum sativum* under different foliar spray and artificial / geo magnetism is as follows: N root + SA foliar spray > S root / N shoot + SA foliar spray > S/N root and N/S shoot + Fe foliar spray > N/S root and S/N shoot + control condition > N root + control condition > S/N root and N/S shoot + control condition > geo magnetism + SA foliar spray > N/S root and S/N shoot + SA foliar spray > S root + control condition > geo magnetism + control condition > S/N root and N/S shoot + SA foliar spray > N/S root and S/N shoot + Fe foliar spray S root / N shoot + Fe foliar spray > N root / S shoot + Fe foliar spray > > N root / S shoot + SA foliar spray > N root / S shoot + control condition > N root + Fe foliar spray > S root / N shoot + control condition > S root + SA foliar spray > S root + Fe foliar spray > geo magnetism + Fe foliar spray.

Like the results of Chl *a*, Chl *b* contents were also positively influenced under different artificial magnetism treatments with Fe and SA foliar supplementation (Fig 2B).

#### 3.2.3. Carotenoids

As far as data of carotenoids is concerned, data was statistically significant (P<0.05). Highest carotenoids were recorded under N root / S shoot treatment with Fe foliar spray; however, minimum carotenoids was observed under S root / N shoot treatment under control condition (Fig 2C).

As per data trend of carotenoids under artificial / geo magnetism and foliar spray, following order was observed: N root / S shoot + iron foliar spray > N/S root and S/N shoot + iron foliar spray > N/S root and S/N shoot + SA foliar spray > S root / N shoot + SA foliar spray > S root / N shoot + iron foliar spray > N/S root and S/N shoot + control condition > N root + iron foliar spray > S root + control condition > N root + SA foliar spray > N root / S shoot + SA foliar spray > S/N root and N/S shoot + SA foliar spray > geo magnetism + SA foliar spray > S root + SA foliar spray > S/N root and N/S shoot + iron foliar spray > N root / S shoot + control condition > geo magnetism + iron foliar spray > S/N root and N/S shoot + control condition > S root + iron foliar condition > N root + control condition > geo magnetism + control condition > S root / N shoot + control condition.

To round up the results of carotenoids it was observed that carotenoid contents enhanced under different artificial magnetism treatment and foliar supplementation while contents of carotenoid remained at lowest under no spray (control set) of all magnetic treatments (i.e., both artificial and geomagnetism) (Fig 2C).

### 3.3. Metabolites

#### 3.3.1. Root soluble sugar

Data of soluble sugar content in roots of pea plant was statistically non-significant (P>0.05). Maximum soluble sugars were recorded in roots of those pea plants which were grown under geomagnetism with Fe foliar spray, whereas minimum soluble sugar content was observed in roots of N root / S shoot magnetism treatment with SA foliar spray (Fig 3A).

**Fig 3:** Effect of different magnetic treatments on the Soluble Sugars Root (A); Shoot (B) of *Pisum sativum* in response to Fe and SA Foliar Spray. The same letters on graphs represent statistically similar effect (P<0.05).

As far as data of soluble sugar in roots is concerned data showed the following trend: Geo magnetism + Fe foliar spray > S root + Fe foliar spray > N root / S shoot + Fe foliar spray > S root / N shoot + Fe foliar spray > N root / S shoot + control condition > N root + Fe foliar spray > N/S root and S/N shoot + control condition > N/S root and S/N shoot + Fe foliar spray > geo magnetism + control condition > N root + control condition > S/N root and N/S shoot + control condition > N/S root and S/N shoot + SA foliar spray > S/N root and N/S shoot + Fe foliar spray > S root + control condition > N root + SA foliar spray > S root / N shoot + control condition > S root + SA foliar spray > S/N root and N/S shoot + SA foliar spray > S root / N shoot + SA foliar spray > geo magnetism + SA foliar spray > N root / S shoot + SA foliar spray.

Considering the above results of soluble sugar content in roots of *Pisum sativum*, it was noted that when plants were grown under different artificial magnetism treatments and Fe foliar spray had greater soluble sugar content while plants with SA foliar applications had the least concentration (Fig 3A).

#### 3.3.2. Shoot soluble sugar

Regarding the data of soluble sugar content in shoots of *Pisum sativum*, the data showed non-significant result among different treatments (P>0.05). Highest soluble sugar content was recorded in shoots under North Root magnetic treatment control condition, whereas lowest soluble sugar content was recorded in shoots of plants grown under geomagnetism with SA foliar application (Fig 3B).

Data of soluble sugar in shoot of pea plant showed the following trend: N root + control condition > N root / S shoot + control condition > S root + control condition > S root / N shoot + control condition > N/S root and S/N shoot + control condition > S/N root and N/S shoot + iron foliar spray > geomagnetism + control condition > N root + iron foliar spray > S/N root and N/S shoot + control condition > S root + iron foliar spray > S root / N shoot + iron foliar spray > N/S root and S/N shoot + iron foliar spray > N root / s shoot + iron foliar spray > geomagnetism + iron foliar spray > S root N shoot + SA foliar spray > S root + SA foliar spray > N root / S shoot + SA foliar spray > N root + SA foliar spray > N/S root and S/N shoot + SA foliar spray > S/N root and N/S shoot + SA foliar spray > geomagnetism + SA foliar spray.

Results of soluble sugar content in shoots revealed that when plants were treated with different artificial magnetism treatments; under control condition (no foliar spray) and Fe spray, the amount of soluble sugar in shoots was at its highest however, foliar spray of SA under all artificial magnetism treatments showed lower soluble sugar content (Fig 3B).

### 3.4. Oxidative stress

#### 3.4.1. Root hydrogen peroxide

Considering data of hydrogen peroxide (H_2_O_2_) concentration in roots of pea plants, statistically non-significant results among different treatments was observed (P>0.05). Highest H_2_O_2_ content was observed in roots of South Root magnetism treatment under control conditions; however, lowest H_2_O_2_ content was observed in roots of N/S root and S/N shoot treatment plants with Fe foliar spray (Fig 4B). Foliar treatment tend to reduce H_2_O_2_ in pea roots under almost all magnetic treatments (about 5–9%).

**Fig 4:** Changes in Oxidative stress Shoot H_2_O_2_ (A), root H_2_O_2_ (B), shoot MDA (C), root MDA (D) parameters of *Pisum sativum* under different magnetic treatments with Fe and SA Foliar Spray.

Data of H_2_O_2_ content in roots of *Pisum sativum* revealed the following trend: S root + control condition > N root / S shoot + control condition > geomagnetism + control condition > N/S root and S/N shoot + SA foliar spray > S/N root and N/S shoot + SA foliar spray > N/S root and S/N shoot + control condition > S root + SA foliar spray > N root / S shoot + Fe foliar spray > S root/ N shoot + Fe foliar spray > S/N root and N/S shoot + Fe foliar spray > S root + Fe foliar spray > N root + control condition > S root / N shoot + SA foliar spray > geomagnetism + Fe foliar spray > N root/ S shoot + SA foliar spray > N root + SA foliar spray > S root / N shoot + control condition > geomagnetism + SA foliar spray > S/N root and N/S shoot + control condition > N root + Fe foliar spray > N/S root and S/N shoot + Fe foliar spray.

To round up the results of H_2_O_2_ in roots of *Pisum sativum* it was revealed that foliar spray of Fe and SA under all magnetic treatment tends to reduce H_2_O_2_ content not to a greater extent but slightly less than the plants with no foliar treatment (Fig 4B).

#### 3.4.2. Shoot hydrogen peroxide

Data recorded for H_2_O_2_ concentration in shoots of *Pisum sativum* showed statistically non-significant results (P>0.05). Maximum H_2_O_2_ content was recorded in shoots of N root / S shoot magnetism under control condition plants while minimum H_2_O_2_ was observed in shoots under N/S root and S/N shoot treatment with Fe foliar application (Fig 4A). Foliar treatment tend to reduce H_2_O_2_ in shoots under almost all magnetic treatments specifically under N/S Root and S/N Shoot magnetic treatment about 7–13%.

Considering data of H_2_O_2_ content in shoots of pea plant under artificial / geo magnetism with Fe and SA foliar spray revealed the following trend: N root / S shoot + control condition > S root + control condition > N root + control condition > geomagnetism + control condition > S/N root and N/S shoot + control condition > S root / N shoot + control condition > N/S root and S/N shoot + control condition > S/N root and N/S shoot + SA foliar spray > N/S root and S/N shoot + SA foliar spray > S root + SA foliar spray. N root / S shoot + SA foliar spray > N root / S shoot + Fe foliar spray > N root + SA foliar spray > S root / N shoot + Fe foliar spray > geomagnetism + Fe foliar spray > geomagnetism + SA foliar spray > S root + Fe foliar spray > N shoot + SA foliar spray > S/N root and N/S shoot + Fe foliar spray > N root + Fe foliar spray > N/S root and S/N shoot + Fe foliar spray.

The overall results of H_2_O_2_ content in shoots of pea revealed that plants when grown under different artificial magnetism treatments and control conditions (no foliar treatment), the amount of H_2_O_2_ in pea plant shoots increased while foliar application of Fe and SA suppressed the accumulation of H_2_O_2_ in plant tissues (Fig 4A).

#### 3.4.3. Root malondialdehyde

As per data of malondialdehyde (MDA) content in roots of pea plant, the data showed statistically non-significant results (P>0.05). Highest MDA contents was observed in roots of those pea plants grown under S root / N shoot magnetism control condition whereas lowest MDA contents was observed in the roots of pea plants under N/S root and S/N shoot magnetic treatment with SA foliar application (Fig 4D). Foliar treatment tend to reduce MDA contents in roots under almost all magnetic treatments specifically under N/S Root and S/N Shoot magnetic treatment about 2–7%.

As far as data of MDA content in roots of pea plant is concerned data revealed the following trend: S root / N shoot + control condition > N root / S shoot + control condition > geo magnetism + control condition > S root + control condition > N root + control condition > N/S root and S/N shoot + iron foliar spray > geomagnetism + iron foliar spray > N root / s shoot + iron foliar spray > S root / N shoot + iron foliar spray > S root + iron foliar spray > S/N root and N/S shoot + iron foliar spray > N root + iron foliar spray > geomagnetism + SA foliar spray > N root / S shoot + SA foliar spray > S root + SA foliar spray > S root / N shoot + SA foliar spray > N root + SA foliar spray > N/S root and S/N shoot + SA foliar spray > S/N root and N/S shoot + SA foliar spray.

Summing up the results of MDA content in roots of pea plant, it was noted that treatments of artificial magnetism under control conditions (no foliar treatment) had elevated levels of MDA in roots while it remain hampered under foliar treatment especially under SA foliar treatment (Fig 4D).

#### 3.4.4. Shoot malondialdehyde

Concerning data of MDA contents in shoot of *Pisum sativum*, data was found to be statistically non-significant (P>0.05) (Fig 4C). Maximum MDA content was observed in shoot of those plants which were grown under N root / S shoot magnetism control conditions; however, lowest MDA was observed in shoots of those plants which were given S root / N shoot treatment with SA foliar spray (Fig 4C).

Data regarding MDA content in shoots of pea plant, under artificial / geo magnetism with Fe and SA foliar spray displayed the following trend: N root / S shoot + control condition > geomagnetism + Fe foliar spray > geomagnetism + control condition > S root /N shoot + control condition > N/S root and S/N shoot + Fe foliar spray > N root + control condition > S root + control condition > S/N root and N/S shoot + control condition > N/S root and S/N shoot + control condition > S/N root and N/S shoot + Fe foliar spray > N root / S shoot + Fe foliar spray > S root + Fe foliar spray > S root / N shoot + Fe foliar spray > N root + Fe foliar spray > geomagnetism + SA foliar spray > S root + SA foliar spray > N root / S shoot + SA foliar pray > N root + SA foliar spray > S/N root and N/S shoot + SA foliar spray > N/S root and S/N shoot + SA foliar spray > S root / N shoot + SA foliar spray.

Concludingly, considering MDA concentration in shoots of pea plant it was observed that under all artificial and geomagnetism treatments the foliar application of SA helped to reduce the level of MDA thus proving its positive role by reducing oxidative stress (Fig 4C).

### 3.5. Nutrients analysis

#### 3.5.1. Root nitrate

As far as data of nitrate content in roots of pea plant is concerned, data showed statistically significant result among different treatments (P<0.05). Maximum nitrate was observed in those roots of pea plant that were under S/N root and N/S shoot magnetism treatment under control, while minimum nitrate was recorded under S root / N shoot treatment with Fe foliar application (Fig 5A).

**Fig 5:** Effect of different magnetic treatments on the Nitrate Root (A), Shoot (B); Iron Root (C), Shoot (D), and Potassium Root (E), Shoot (F), content of *Pisum sativum* in response to Fe and SA Foliar Spray. The same letters on graphs represent statistically similar effect (P<0.05).

Data trend regarding nitrate content in roots of *Pisum sativum*, showed the following trend: S/N root N/S shoot + control condition > geo magnetism + control condition > N/S root S/N shoot + control condition > S root / N shoot + control condition > geo magnetism + SA foliar spray > N/S root S/N shoot + SA foliar spray > S/N root N/S shoot + SA foliar spray > N root + control condition > S root + SA foliar spray > N root / S shoot + control condition > N root / S shoot + SA foliar spray > S root / N shoot + SA foliar spray > S root + control condition > N root + SA foliar spray > N root + Fe foliar spray > S/N root N/S shoot + Fe foliar spray > S root + Fe foliar spray > geo magnetism + Fe foliar spray > N/S root S/N shoot + Fe foliar spray > N root / s shoot + Fe foliar spray > S root / N shoot + Fe foliar spray.

In a nutshell, considering the above results, it was observed that nitrate in roots of *Pisum sativum* increased when plant was applied with different artificial magnetism treatments under control condition (no foliar treatment) (Fig 5A).

#### 3.5.2. Shoot nitrate

Regarding nitrate content in shoots of pea plant, it was observed that the data was statistically significant (P<0.05). Maximum nitrate was observed in shoots of N root / S shoot treatment plants under control condition, whereas least nitrate was observed under S root / N shoot magnetism with Fe foliar spray (Fig 5B).

Data of nitrate in shoot showed the following trend under artificial / geo magnetism with Fe and SA foliar spray: N root / S shoot + control condition > S/N root and N/S shoot + control condition > S/N root and N/S shoot + SA foliar spray > N/S root and S/N shoot + control condition > geo magnetism + control condition > N root + control condition > geo magnetism + SA foliar spray > S root / N shoot + control condition > N/S root and S/N shoot + SA foliar spray > S root / N shoot + SA foliar spray > S root + SA foliar spray > N root / S shoot + SA foliar spray > S root + control condition > N root + SA foliar spray > N root + Fe foliar spray > S root + Fe foliar spray > N root / S shoot + Fe foliar spray > S/N root and N/S shoot + Fe foliar spray > geo magnetism + Fe foliar spray > N/S root and S/N shoot + Fe foliar spray > S root / N shoot + Fe foliar spray.

The trend of nitrate content in shoots of pea plants was similar to those of nitrate root. Nitrate contents in shoots increased when given the artificial magnetism treatments under control conditions and least nitrate contents was observed under Fe foliar application (Fig 5B).

#### 3.5.3. Root iron

As far as data of iron (Fe) content in roots of *Pisum sativum* is concerned, it is found to be statistically significant (P<0.05). Maximum Fe content was observed in roots of those plants which were grown under S root / N shoot magnetism + Fe foliar spray while minimum Fe was observed under S/N root and N/S shoot treatment with SA and Fe foliar spray (Fig 5C).

Data of iron content in roots of *Pisum sativum* showed the following trend under artificial / geo magnetism with Fe and SA foliar spray: S root / N shoot + iron foliar spray > S root / N shoot + SA foliar spray > geomagnetism + iron foliar spray > geomagnetism + SA foliar spray > N root + SA foliar spray > S/N root and N/S shoot + control condition > S root + SA foliar spray > S root + iron foliar spray > N root + iron foliar spray > N root / S shoot + control condition > N root / S shoot + SA foliar spray > N root / S shoot + iron foliar spray > S root / N shoot + control condition > N/S root and S/N shoot + control condition > N/S root and S/N shoot + SA foliar spray > N/S root and S/N shoot + iron foliar spray > N root + control condition > geomagnetism + control condition > S root + control condition > S/N root and N/S shoot + iron foliar spray = S/N root and N/S shoot + SA foliar spray.

Considering the results of Fe content in roots of *Pisum sativum* under foliar spray and artificial magnetism treatments, it was observed that SA and Fe foliar applications helped in improving the amount of Fe under different magnetism treatments (Fig 5C).

#### 3.5.4. Shoot iron

Regarding the data of Fe in shoots of *Pisum sativum* data showed statistical significance among different treatments (P<0.05). Maximum iron content was observed in shoots of those *Pisum sativum* which were grown under S/N root and N/S shoot magnetism with Fe foliar spray; however, minimum Fe content was observed with North root magnetism treatment under control condition (Fig 5D).

Data regarding Fe content in shoots of pea plant, revealed the following trend: S/N root and N/S shoot + Fe foliar spray > N root + SA foliar spray > S/N root and N/S shoot + SA foliar spray > N/S root and S/N shoot + Fe foliar spray > S root / N shoot + SA foliar spray > geomagnetism + SA foliar spray > S root / N shoot + Fe foliar spray > N root / S shoot + SA foliar spray > N/S root and S/N shoot + SA foliar spray > S root / N shoot + control condition > S/N root and N/S shoot + control condition > S root + SA foliar spray > geomagnetism + Fe foliar spray > S root + Fe foliar spray > N/S root and S/N shoot + control condition > N root / S shoot + control condition > geomagnetism + control condition > N root + Fe foliar spray > N root / S shoot + Fe foliar spray > S root + control condition > N root + control condition.

Correlating the results of Fe content in roots with shoots it was observed that in both, trend was almost similar. Fe and SA enhanced the amount of iron in shoots under different artificial magnetism treatments (Fig 5D).

#### 3.5.5. Root potassium

Considering data of potassium (K^+^) in roots of pea plant it was observed that the data was statistically significant (P<0.05). Highest potassium was noted in roots of plants under geomagnetism control condition, whereas lowest potassium was recorded in roots under S root / N shoot magnetism under control condition (Fig 5E).

As far as data of K^+^ in roots of *Pisum sativum* is concerned under artificial / geo magnetism with Fe and SA foliar spray revealed the following trend: Geomagnetism + control condition > S root + control condition > S/N root and N/S shoot + SA foliar spray > S root / N shoot + iron foliar spray > N root + control condition > n root / S shoot + SA foliar spray > geomagnetism + iron foliar spray > S root / N shoot + SA foliar spray > N/S root and S/N shoot + SA foliar spray > N root + iron foliar spray > geomagnetism + SA foliar spray > N/S root and S/N shoot + control condition > S root + iron foliar spray > S root + SA foliar spray > N root + SA foliar spray > N/S root and S/N shoot + iron foliar spray > N root / S shoot + iron foliar spray > S/N root and N/S shoot + control condition > N root / S shoot + control condition > S/N root and N/S shoot + iron foliar spray > S root / N shoot + control condition.

Considering the overall results of potassium in roots of pea plant, it was observed that Fe and SA foliar spray under artificial magnetism treatments increased the level of potassium in roots (Fig 5E).

#### 3.5.6. Shoot potassium

As per data of K^+^ in shoots of *Pisum sativum*, it revealed to be statistically significant (P<0.05). Highest potassium content was observed in shoots of those pea plants, which were treated with S root / N shoot magnetism with SA foliar spray whereas the least potassium was observed in shoots of those plants which were grown with N root / S shoot magnetism under control conditions (Fig 5F).

Data of potassium in shoots of pea plant showed the following trend: S root / N shoot + SA foliar spray > geomagnetism + SA foliar spray > S/N root and N/S shoot + Fe foliar spray > N/S root and S/N shoot + SA foliar spray > N/S root and S/N shoot + Fe foliar spray > S/N root and N/S shoot + SA foliar spray > N root / S shoot + SA foliar spray > N root + SA foliar spray > S root / N shoot + Fe foliar spray > S root + SA foliar spray > geomagnetism + Fe foliar spray > N root / S shoot + Fe foliar spray > N root + Fe foliar spray > S root + Fe foliar spray > geomagnetism + control condition > N/S root and S/N shoot + control condition > N root + control condition > S/N root and N/S shoot + control condition > S root + control condition > S roots / N shoot + control condition > N root / S shoot + control condition.

In a nutshell, overall results of potassium in shoots of *Pisum sativum*, revealed that the level of potassium in shoots increased under different artificial magnetism treatments and Fe/SA foliar supplementation (Fig 5F).

## 4. Discussion

Several studies have shown that the applications of magnetic treatments have positive influence on different morphological parameters like root length, shoot length, number of leaves, leaf area of plant, root fresh weight, shoot fresh weight, root dry weight, shoot dry weight [46–48]. It has been observed in present research that when the artificial magnetic treatment has been applied to pea plants, there was an overall enhancement in different morphological parameters like root length (63.41%), shoot length (35.29%), leaf area per plant (64.82%), over geomagnetism treated plants. Our results are consistent with those of [3] who reported that effects of magnetic field have shown positive effects on germination, growth of soybean under salinity stress. Magdalena et al. [49] documented that 130 mT magnetic field treatment increases shoot length and shoot weights in Lupin. Omid [50] elaborated that magnetized water had positive impact on growth and yield of cowpea plants. Bukhari et al. [48] further validates the findings that magnetic field treatment stimulates growth and development of sunflower seedlings. López-Millán et al. [51] reported that exogenous application of Fe is very beneficial in the enhancement of total mass of the whole plant but when Fe is deficient, it limits growth of root and shoot, leaf area and No. of leaves was observed in many plant species. In present research, it was observed that under different combinations of artificial magnetism treatment with Fe foliar spray have positively influenced several growth parameters. Exogenous Fe foliar spray enhanced root length, shoot length and shoot dry weight under specific magnetic treatment (Fig 1A, 1B and 1H). Our results are in agreement with the findings of Rawashdeh and Sala [52] who documented that foliar supplementation of Fe alone or in combination with B (Boron) significantly increased wheat root and seedling length along with fresh and dry weights of shoot and root compared to control wheat seedlings. Several researches validates that supplementation of Fe increases growth and yield of crops [36, 37]. While considering the results of root fresh and dry weights, it was observed that SA foliar treatment tend to improves under different magnetic treatments (Fig 1E and 1H). Correspondingly, Yadav et al. [28] reported an increase in plant height and grain yield of wheat with better RWC%, with SA foliar supplementation under salinity and drought stress.

Moreover, North Root magnetic treatment (no foliar treatment/control) had maximum SFW and Leaf area plant^-1^ (Fig 1F and 1D), whereas South Root magnetic treatment under control and SA foliar treatment had longest roots and maximum RFW respectively (Fig 1A and 1E) suggesting that North Root treatment enhances leaf area/plant thereby increasing plant shoot fresh weights however South magnetic treatment promotes root development. Smith et al. [53] corroborates that root growth is quite more sensitive to magnetic fields as compared to shoots. Aladjadjiyan [54] reported that the energy of magnetic field strength had stimulative effects on different physiological and developmental attributes of the plants. He reported in his research that magnetic field energy had a positive impact on some paramagnetic atoms and photosynthetic pigments in the plant cells. Which is quite evident in present research as it was noted in the case of chlorophyll *a*, it remain highest in control conditions (no foliar treatment) of various artificial magnetic treatments (Fig 2A). Literature supports our finding that Chl increases under magnetic field treatment as reported in potato [55] and maize [56]. However, application of SA foliar spray increased the contents of chlorophyll *b* in response to various artificial magneti treatment (Fig 2A and 2B) which is endorsement of Yusuf et al. [29] who reported that SA has positive effects on the activity of Rubisco (ribulose 1, 5 bisphosphate) as well as on chlorophyll contents. However, Yadav et al. [28] found an increase in total Chl contents, with SA foliar treatment. Moreover, amount of carotenoids was recorded at its maximum with Fe foliar spray (Fig 2C) as reported by Sen and Alikamanoglu [11] that magnetic treatment increases carotenoid content in wheat. Similar findings were also reported by Selim and El-Nady [6] in tomato under magnetic treatment in response to drought stress. Nilimesh et al. [57] documented that presowing magnetic field treatment increases carotenoid content in chickpea under soil moisture stress. Furthermore it is important to note that North Root treatment tend to have maximum chlorophyll contents as compared to other magnetism treatment.

Furthermore, several researchers documented that treatments of magnetism have been reported to be quite useful in enhancing primary and secondary metabolites of different plant species. As it has been studied by Luna et al. [58] that continuous treatment of magnetic field increased the accumulation of lipids, proteins, and carbohydrates at exponential growth phase whereas enhanced the accumulation of lipids at stationary phase. One of the essential osmotic solutes i.e. Soluble sugars increases by the foliar application of SA [59]. The application of Salicylic acid (SA) enhances the content of soluble sugar of tomato plant which were exposed to salt stress due to the properties of soluble sugar being compatible solute highly accumulated in plant tissues exposed to abiotic stress [25]. Considering the results of shoot soluble sugars content of *Pisum sativum* it was observed that it increased under different magnetic treatments which is in consistent to the results of [9] who documented that magnetic treatment increases solule sugars in plants under salt stress. Soluble sugars were specially higher under foliar treatment of Fe (Fig 3B) Contrarily, Abdoli et al. [26] reported that under SA foliar treatment the concentration of soluble sugar increases under salt stress. Accumulation of soluble sugar act as an important role in the defensive mechanisms of plant. Therefore, it is inferred that the exogenous application of SA can improve the osmoregulation in plants [18]. However, Mohamed et al. [60] reported that the contents of soluble sugar increases under foliar application of Fe. Furthermore, Deamici et al. [61] reported that magnetic treatment increases overall carbohydrate content by 24.8%.

Oxidative stress arises as a consequence of environmental stress and against the attack of different pathogens leading to the generation of H_2_O_2_, hydroxyl radicals (ROS Species), and MDA content [62]. Abdollahi et al. [46] quoted that foliar treatments of SA and iron oxide positively affect oxidative stress antioxidant enzymes that include polyphenol oxidase, CAT, POD, and SOD. SA as foliar treatment tend to increase POD, SOD, CAT, soluble sugars, glycine betaine, protein, relative water content, while decrease H_2_O_2_, O2^•−^, and MDA. However, the current study noted that different combinations of artificial magnetism treatments with Fe and SA foliar spray have been beneficiary in decreasing the level of oxidative stress (Fig 4A–4D). It was observed that when pea plant under N/S Root and S/N Shoot magnetism and Fe foliar spray reduced the level of hydrogen peroxide in the shoot of *Pisum sativum* (Fig 4A). Whereas in the case of MDA it was observed that SA foliar treatment both in shoot and root reduced the level of MDA under all artificial magnetic treatment (Fig 4C and 4D). Chen et al. [63] documented similar results as a decrease in MDA and H_2_O_2_ content in mungbean under 600 mT magnetic field treatment was observed. Contrarily, Abdollahi et al. [10] documented that magnetized field increases MDA content in *Citrus aurantifolia* healthy and infected plants as compared to control plants.

Noran et al. [64] reported that magnetic field treatment decreased the downward movements of calcium, potassium, iron, nitrogen, sodium, and magnesium as magnetic field treatment enhances the concentration of these nutrients in plants as compared to control conditions. It has been observed that magnetic treatment positively affects the ion concentration, free radical movements, and electric charges without inducing any changes in studied that magnetic field treatments effectively reduce the pH of the soil resulting in the highest uptake of nutrients from the soil, ultimately increasing the level of calcium and potassium. In present research nutrients (Fe, K, and NO_3_^-^) tend to increase under various magnetic treatments and impact of foliar treatment. Our findings are in agreement it the findings of Shahin et al [65] documented that magnetic treatment of irrigation water significantly increases nutrient absorption N,P, K. Fe, Cu, Zn and Mn in *Glycine max*. Similarly Esitken and Turan [66] reported an increase in fruit yield of strawberry under alternative magnetic treatment with an increase in mineral nutrients, i.e., N, Ca, Fe, Mn, K, and Zn. Moreover, SA foliar treatment effect was more pronounced in shoot as compared to roots as; K, NO_3_^-^, and Fe were higher in all respective magnetic treatments compared to control (no foliar spray), and Fe supplemented plants (Fig 5A–5F). Souri and Tohidloo [67] documented that foliar treatment of SA significantly increased; leaf Fe and K under salinity stress. Furthermore, nitrate accumulation both in shoot and root gets limited under Fe foliar supplementation (Fig 5A and 5B). These results suggested that an increase in Fe concentration causes a reduction in nitrate content of shoot while an increase was observed in Cu, Mn, P, and Na contents. The illustration makes it clear that excessive concentration of Fe was reported to minimize the concentration of Mn, Zn, and Na in both root and shoot of pea under stress conditions such as salinity.

In a nutshell, different treatments of artificial magnetism had a strong impact on the growth and physiology of pea plant; moreover, various attributes (both growth and physiological) endorsed the foliar supplementation of Fe and SA under magnetic treatments. Therefore, in the near future, omics-based studies could be carried out with under artificial magnetism to reveal the molecular mechanisms associated with hormones and magnetism treatments in crop plants [68].

## 5. Conclusion

Seeds treated with a magnetic field before sowing improve the growth and productivity of crops. Exposing *Pisum sativum* to artificial magnetism treatments in response to Fe and SA foliar application showed encouraging effects on plant growth as it improved several morphological attributes in comparison to geomagnetism. Results also showed positive effects of artificial magnetism along with foliar supplementation of Fe and SA that enhanced photosynthetic pigments, accumulation of soluble sugars and nutrients (Fe, K, and NO_3_^-^) in pea plant, thus suggesting the positive interaction of foliar spray to magnetism. In general, using different kinds of chemicals for better crop growth and yield has been a successful practice, but it is quite detrimental to the environment and soil. Using magnetic fields as a pre-sowing treatment with plant growth regulators can be safe and eco-friendly agricultural practices as compared to using chemicals. Moreover, understanding the positive and negative effects of different magnetic fields will help the researchers to understand the evolutionary changes in plants due to magnetic fields for future exploration. Furthermore, detailed proteomic and genomic analyses of plants treated with various magnetic treatments would further help to understand and explore the effect of magnetic fields on various plants.

## Supporting information

S1 Data (RAR)

S1 File (DOCX)
